The article "Relationship between Dynamic Changes of Microcirculation Flow, Tissue Perfusion Parameters, and Lactate Level and Mortality of Septic Shock in ICU" was published in 2022. Journal: Contrast Media Mol Imaging.

# Relationship between Dynamic Changes of Microcirculation Flow, Tissue Perfusion Parameters, and Lactate Level and Mortality of Septic Shock in ICU

**DOI:** 10.1155/2022/1192902

**Published:** 2022-10-07

**Authors:** Xuebing Yang, Yaqing Zhou, Aiming Liu, Zunguo Pu

**Affiliations:** Department of Critical Care Medicine, Affiliated Hai'an Hospital of Nantong University, Hai'an County, Nantong, Jiangsu Province 226600, China

## Abstract

**Background:**

Septic shock is a common clinical critical disease with high mortality, hemodynamic instability, and easy to be complicated with multiple organ failure. The rapid progress of the patient's condition poses a serious threat to patient's safety.

**Aim:**

To investigate the relationship between the dynamic monitoring of microcirculation perfusion parameters and blood lactic acid level and the prognosis of patients with infection shock in ICU.

**Methods:**

A total of 104 patients with septic shock admitted to ICU of Affiliated Hai'an Hospital of Nantong University from February 2018 to June 2021 were selected for clinical research. According to the survival situation of patients after 28 days of treatment, they were divided into the death group (*n* = 48) and the survival group (*n* = 56). The central venous-arterial carbon dioxide partial pressure difference (Pcv-aCO2), the ratio of central venous-arterial carbon dioxide partial pressure difference to arterial central venous oxygen content difference (Pcv-aCO2/Ca-cvO2), and blood lactic acid level were retrospectively analyzed and compared between the two groups on the first, third, and seventh days after admission to ICU. The odds ratio (OR) of three indexes affecting the prognosis of patients with septic shock was analyzed by univariate and multivariate mathematical models, and the value of three indexes in predicting the prognosis of patients was analyzed by receiver operating curve (ROC).

**Results:**

Pcv-aCO2 and lactic acid in the death group were higher than those in the survival group on the 1st, 3rd, and 7th day of ICU stay (*P* < 0.05). The Pcv-aCO2/Ca-cvO2 of the death group was higher than that of the survival group on the 3rd and 7th day of ICU stay (*P* < 0.05). Logistic model results showed that age, SOFA score, APACHE II score, the number of multiple organ failure (MODS), intracranial infection, the increase of Pcv-aCO2, Pcv-aCO2/Ca-cvO2, and the increase of lactic acid were independent risk factors for death in patients with septic shock (OR values were 1.519, 1.808, 1.781, 1.912, 2.069, 1.848, 1.781, and 1.642, respectively, *P* < 0.05). The results showed that the AUC value of Pcv-aCO2 in predicting death was 0.943, and the sensitivity and specificity were 93.72% and 83.09%, respectively. The AUC value of Pcv-aCO2/Ca-cvO2 for predicting death was 0.887, and the sensitivity and specificity were 81.63% and 77.56%, respectively. The AUC value of lactic acid in predicting death of patients was 0.825, and the sensitivity and specificity were 71.66% and 82.09%, respectively.

The article "Relationship between Dynamic Changes of Microcirculation Flow, Tissue Perfusion Parameters, and Lactate Level and Mortality of Septic Shock in ICU" was published in 2022. Journal: Contrast Media Mol Imaging.

**Conclusion:**

Changes of microcirculation flow tissue perfusion parameters and blood lactic acid level changes are closely related to the prognosis of patients with septic shock, which is of great value in the evaluation of the prognosis of patients with septic shock.

## 1. Introduction

Septic shock is a common clinical critical illness, with high mortality, hemodynamic instability, easy to merge multiple organ failure, and other characteristics. The patient's condition progresses rapidly and poses a serious threat to the safety of patients. The basic pathological features of the patients were systemic vascular dilatation and increased capillary permeability, showing insufficient circulating blood volume, reduced tissue perfusion, and systemic metabolic disorder [1]. Accurate evaluation of tissue perfusion for patients with septic shock is of great significance for guiding clinical treatment, and the prognosis of patients' needs to be evaluated. The changes of central venous-arterial carbon dioxide concentration can reflect the perfusion state of microcirculation flow tissue. Pcv-aCO2 and Pcv-aCO2/Ca-cvO2 are commonly used clinical indicators, which can reflect the oxygen metabolism state at the cellular level and understand the hemodynamic changes. Lactic acid is a commonly used index for clinical evaluation of tissue hypoxia and ischemia. There is a certain correlation between the concentration of blood lactic acid and the severity of the disease [2]. In this study, patients with septic shock were taken as the research object to analyze the relationship between the microcirculation perfusion parameters, blood lactic acid level changes, and the prognosis of patients, so as to find reliable indicators to evaluate the microcirculation perfusion of patients with septic shock. The report is as follows.

*Core tips*: shock is a common and critical disease in clinical practice, with diverse and complex etiology, difficult treatment, and poor prognosis. Shock, as a name for a syndrome, can describe the occurrence and development of circulatory failure. It is very important to monitor shock. Early detection and early intervention at the same time pay attention to the integrity, and continuity of shock intervention has important value to improve the prognosis of patients. Therefore, reasonable selection of indicators with good sensitivity and specificity is of great significance to the treatment and prognosis of shock. Traditionally, the microcirculatory perfusion index of patients is evaluated with central venous pressure and peripheral perfusion index, but there are many influencing factors, the specificity is not high, and it is easily influenced by subjective factors. Central venous-arterial carbon dioxide partial pressure difference can reflect the tissue perfusion of microcirculation flow. The analysis of local tissue blood flow and cellular oxygen metabolism can guide clinical treatment and evaluate prognosis. Lactic acid is the product of anaerobic digestion. Generally, the body has shown insufficient perfusion before hemodynamic changes, and oxygen transport and utilization are hindered. Therefore, the monitoring of lactic acid can reflect the development and prognosis of patients with septic shock. In this study, patients with septic shock were selected as the research objects to analyze the relationship between the changes of microcirculation flow tissue perfusion parameters and blood lactic acid level and the prognosis of patients.

The article "Relationship between Dynamic Changes of Microcirculation Flow, Tissue Perfusion Parameters, and Lactate Level and Mortality of Septic Shock in ICU" was published in 2022. Journal: Contrast Media Mol Imaging.

## 2. Materials and Methods

### 2.1. General Information

104 patients with septic shock admitted to ICU of Affiliated Hai'an Hospital of Nantong University from February 2018 to June 2021 were selected for clinical study. According to the survival situation of patients after 28 days of treatment, they were divided into death group (48 cases) and survival group (56 cases).

Inclusion criteria are as follows: (1) the age of the patients ranged from 19 to 79 years. (2) Diagnostic criteria for patients with septic shock refer to the criteria in the Guidelines for Emergency Diagnosis and Treatment of Sepsis/Septic Shock in China 2018 [3]. (3) Patients stay in ICU more than one week, the test data is complete. (4) The research program meets the requirements of the medical ethics expert group in our hospital. Exclusion criteria are as follows: (1) patients without central venous catheter. (2) Patients with long-term use of immunosuppressants or regulators due to disease. (3) End-stage cancer patients. (4) Pregnant women or lactation women. (5) Epilepsy, psychosis, etc.

### 2.2. Indicator Detection

The general data of patients were collected, and the age, sequential organ failure score (SOFA), acute physiology and chronic health evaluation II (APACHE II), ICU hospitalization time, number of multiple organ failure (MODS), mean artery pressure (MAP), 24h urine volume, and other related data were recorded. At the same time, the prognosis of patients was recorded, and the data were input into the computer system for analysis.

The article "Relationship between Dynamic Changes of Microcirculation Flow, Tissue Perfusion Parameters, and Lactate Level and Mortality of Septic Shock in ICU" was published in 2022. Journal: Contrast Media Mol Imaging.

The SOFA score consists the following 6 parts: respiration, coagulation, liver, cardiovascular, central nervous system, and renal, and the higher the score, the worse the prognosis. The APACHE II scoring system consists the acute physiology score, age score, and chronic physiology score, and the higher the score, the worse the prognosis.

*Instrument*: Danish Raydu company blood gas analyzer, model AL800 FLEX, was employed. Collect 1 ml of peripheral artery, central venous blood of each patient, gently rub the syringe in the palm back and forth 5-6 times, click the blood gas analyzer screen sample key, connect the syringe and port, according to the instrument prompt input patient information, and check the parameters. The calculation formula was Pcv−aCO2 = PcvCO2−PaCO2; ca-cvO2 = CaO2-CcvO2 = 1.36 × Hb × (SaO2-SvO2) ml/dl.

The fasting venous blood of 3 ml was extracted and centrifuged at 2000 r/min for 30 min. The instrument selected Hitachi 7600 i automatic immune biochemical analyzer. The blood lactate concentration was determined by using enzyme-linked immunosorbent assay. The serum albumin concentration was determined by using electrochemical analysis. The kit was provided from Nanjing Jiancheng Biological Products Co, Ltd.

### 2.3. Statistical Processing

The measurement indexes such as Pcv-aCO2, Pcv-aCO2/Ca-cvO2, and lactic acid test of the two groups of patients collected in this study were subjected to normal distribution test, which were in line with the approximate normal distribution or normal distribution, expressed as ($\bar{x}$ ± *s*), and compared between the two groups by *t*-test. *χ*2 test or Fisher exact test was used for comparison between groups of nongrade counting data; the receiver operating curve (ROC) was used for the prediction model. Multivariate analysis model using logical data analysis method; data processing using professional SPSS21.0 software, test level *α* = 0.05.

## 3. Results

### 3.1. Comparison of Pcv-aCO2, Pcv-aCO2/Ca-cvO2, and Lactic Acid between the Death Group and Survival Group

Pcv-aCO2 and lactic acid in the death group were higher than those in the survival group on the 1st, 3rd, and 7th day of ICU stay (*P* < 0.05). The Pcv-aCO2/Ca-cvO2 of the death group was higher than that of the survival group on the 3rd and 7th day of ICU stay (*P* < 0.05). The Pcv-aCO2/Ca-cvO2 on the 1st day of ICU stay was not significantly different between the death group and the survival group (*P* > 0.05) (Table 1).

### 3.2. Comparison of Single Factor Analysis between the Death Group and Survival Group

The age, SOFA score, APACHE II score, ICU length of stay, and the number of MODS in the death group were higher than those in the survival group, and the proportion of patients with intracranial infection was higher than that in the survival group (*P* < 0.05). Serum albumin, MAP, and 24 h urine volume in the death group were lower than those in the survival group (*P* < 0.05). The BMI, mechanical ventilation time, gender, smoking, drinking, and reason for admission to ICU were not significantly different between the death group and the survival group (*P* > 0.05) (Table 2).

The article "Relationship between Dynamic Changes of Microcirculation Flow, Tissue Perfusion Parameters, and Lactate Level and Mortality of Septic Shock in ICU" was published in 2022. Journal: Contrast Media Mol Imaging.

### 3.3. Multivariate Analysis of Prognostic Factors in Patients with Septic Shock

The death of patients with septic shock was taken as the dependent variable, and the age, SOFA score, APACHE II score, ICU length of stay, the number of MODS, serum albumin, MAP, 24-hour urine volume, Pcv-aCO2, Pcv-aCO2/Ca-cvO2, and lactic acid determination values on the third day of ICU stay were taken as independent variables in the univariate analysis. The results of the logistic model showed that the increase of age, SOFA score, APACHE II score, the number of MODS, intracranial infection, the increase of Pcv-aCO2 on the third day of ICU stay, the increase of Pcv-aCO2/Ca-cvO2, and the increase of lactic acid determination values were the independent risk factors for the death of patients with septic shock (OR values were 1.519, 1.808, 1.781, 1.912, 2.069, 1.848, 1.781, and 1.642, respectively, and all of the -values were less than 0.05) (Table 3).

### 3.4. ROC Curve Analysis of Pcv-aCO2, Pcv-aCO2/Ca-cvO2, and Lactic Acid in Predicting Death of Patients

ROC curve was drawn by Pcv-aCO2, Pcv-aCO2/Ca-cvO2, and lactic acid on the third day of ICU admission. The results showed that the AUC value of Pcv-aCO2 in predicting death was 0.943, and the sensitivity and specificity were 93.72% and 83.09%, respectively. The AUC value of Pcv-aCO2/Ca-cvO2 for predicting death was 0.887, and the sensitivity and specificity were 81.63% and 77.56%, respectively. The AUC value of lactic acid in predicting death of patients was 0.825, and the sensitivity and specificity were 71.66% and 82.09%, respectively (Table 4, Figure 1).

## 4. Discussion

Septic shock, also known as sepsis, is a serious clinical syndrome. The hemodynamic fluctuation of patients is large, and the disease progresses rapidly. The mortality rate of septic shock worldwide is high. The number of patients with sepsis is more than 30 million each year, and the mortality rate is 20%, which has a serious impact on the life safety of patients [3]. At present, it is considered that patients with septic shock have abnormal vasoconstriction function and changes in blood flow distribution, showing a low blood volume state. Insufficient perfusion will lead to ischemia and hypoxia of tissues and organs. Among them, insufficient oxygen supply to tissues and dysfunction of oxygen utilization are important causes of tissue cell hypoxia. Therefore, monitoring the hemodynamics of patients is of great significance for evaluating the prognosis of patients [4, 5].

The article "Relationship between Dynamic Changes of Microcirculation Flow, Tissue Perfusion Parameters, and Lactate Level and Mortality of Septic Shock in ICU" was published in 2022. Journal: Contrast Media Mol Imaging.

At present, it is considered that blood pressure reduction is not sensitive in the evaluation of septic shock, and the body can maintain blood pressure by compensatory mechanism in the early stage, so microcirculation perfusion index has been applied in clinical practice in recent years. In this study, Pcv-aCO2 and Pcv-aCO2/Ca-cvO2 in the death group were significantly increased after admission to ICU. Pcv-aCO2 can reflect the oxygen metabolism in patients, which generally referred to the tension formed by physical dissolution of carbon dioxide in central venous blood and arterial blood. The content of carbon dioxide in blood was almost linear with the partial pressure of carbon dioxide, and there was no saturation point. When the body hemodynamics was stable, the partial pressure of carbon dioxide in central venous blood and arterial blood was close. Once the index was increased, it indicated that tissue perfusion was insufficient [6, 7]. Pcv-aCO2/Ca-cvO2 reflects respiratory entropy. The concentration of carbon dioxide formed by aerobic metabolism decreases after tissue hypoxia. The body forms a large number of acidic substances under anaerobic metabolism and forms a large amount of carbon dioxide under the action of blood buffering system. Therefore, the increase in Pcv-aCO2/Ca-cvO2 suggested that anaerobic metabolism increases [8, 9].

In this study, the concentration of lactic acid in the dead patients was significantly higher than that in the survival group. The formation of lactic acid reflects the increase of anaerobic metabolism in the human body and the mismatch between oxygen transport and consumption. The increase of lactic acid has an impact on the stability of the internal environment in the body, especially on the heart function and the process of oxygen metabolism in the human body. It will aggravate the state of tissue hypoxia. The combination of endotoxin and receptor in patients with severe septic shock will cause increased activation of inflammatory factors, and inflammatory mediators will mediate biochemical cascade and aggravate circulatory disorders in the body [10]. Some studies have found that the uptake and utilization of oxygen in human tissues have changed after severe infection. The functional changes of microcirculation and tissue metabolic dysfunction exist in the whole process of infection. Inflammatory reaction leads to mitochondrial dysfunction, which also affects the utilization of oxygen by cells. Finally, hypoxia and metabolic dysfunction in tissues are aggravated [11]. In this study, ROC curve was drawn and it was found that the measured values of Pcv-aCO2, Pcv-aCO2/Ca-cvO2, and lactic acid had certain predictive value for the death of patients with septic shock, with the AUC values of 0.943, 0.887, and 0.825, respectively. These results also illustrate the above mechanisms.

The article "Relationship between Dynamic Changes of Microcirculation Flow, Tissue Perfusion Parameters, and Lactate Level and Mortality of Septic Shock in ICU" was published in 2022. Journal: Contrast Media Mol Imaging.

This study also analyzed the risk factors of death in patients with septic shock. It was found that age, SOFA score, APACHE II score, MODS number, and intracranial infection were risk factors for death in patients with septic shock. APACHE II score is of great significance in the analysis of the severity of illness and prognosis evaluation of critically ill patients. The higher the score is, the more serious the patient is. Therefore, it can reflect the severity of illness in patients with septic shock. The higher the score is, the worse the treatment effect is and the higher the risk of death is [12–15]. The increase of SOFA score often indicates more and more serious organ failure, which will affect the final clinical outcome of patients. The increase of age, the number of MODS, intracranial infection, and other factors will affect the clinical treatment effect of patients. The older the patient, the more pronounced the decline in immune function The more the number of organs affected, the more serious the patient's condition is, the more affected organs are, and the risk of death increases [16, 17]. However, there were differences in the analysis of age reported in the past. Considering that the increase of age will lead to the increase of APACHE II score of patients, and generally elderly patients have more comorbidities and complications, these factors partially offset the impact of age on mortality, which is inconsistent with the results of this study [18–20].

This study analyzed the influencing factors of prognosis in patients with septic shock and provided a certain value for clinical positive evaluation of prognosis. Using microcirculation flow perfusion parameters and blood lactic acid level to evaluate prognosis can reflect the changes of organ function in patients more timely and accurately. However, the number of cases included in the study is small, and it is a single-center study. Small sample size will lead to selective bias. Moreover, patients are all ICU patients, most of whom are transferred from the general ward. Some patients were failed to be treated according to the cluster process at the first time when shock occurs, which might affect the accuracy of the results. Therefore, it is necessary to further carry out large sample size and prospective randomized study to demonstrate the results.

The article "Relationship between Dynamic Changes of Microcirculation Flow, Tissue Perfusion Parameters, and Lactate Level and Mortality of Septic Shock in ICU" was published in 2022. Journal: Contrast Media Mol Imaging.

In summary, the changes of microcirculation flow tissue perfusion parameters and blood lactic acid level are closely related to the prognosis of patients with septic shock, which is of great value in the evaluation of the prognosis of patients with septic shock.

The study is approved by ethics committee of Hai'an Hospital Affiliated to Nantong University.

## Figures and Tables

**Figure 1:** ROC curve of Pcv-aCO_2_, Pcv-aCO_2_/Ca-cvO_2_, and lactate values in predicting the death of patients.

**Table 1:** Comparison of Pcv-aCO2, Pcv-aCO2/Ca-cvO2, and lactate between the death group and survival group ($\bar{x}$±*s*).

Index	Group	Day 1	Day 3	Day 7
Pcv-aCO_2_ (mmHg)	Death group (*n* = 48)	5.74 ± 1.62	7.98 ± 1.55	6.43 ± 1.65
	Survival group (*n* = 56)	3.40 ± 1.34	4.41 ± 1.73	3.28 ± 1.22
	*T*	8.062	11.003	11.166
	*P*	0.000	0.000	0.000

Pcv-aCO_2_/Ca-cvO_2_ (mmHg/mL)	Death group (*n* = 48)	2.26 ± 0.63	3.72 ± 0.84	2.81 ± 0.70
	Survival group (*n* = 56)	2.07 ± 0.70	2.45 ± 0.71	1.69 ± 0.55
	*T*	1.445	8.357	9.131
	*P*	0.152	0.000	0.000

Lactic acid (mmol/L)	Death group (*n* = 48)	4.01 ± 1.43	5.52 ± 1.62	3.76 ± 1.10
	Survival group (*n* = 56)	2.47 ± 0.69	3.31 ± 0.82	2.82 ± 0.66
	*T*	7.150	8.962	5.368
	*P*	0.000	0.000	0.000

**Table 2:** Univariate analysis results.

Normal information	Death group (*n* = 48)	Survival group (*n* = 56)	*t*/*χ*^2^	*P*
Age (years)	68.2 ± 7.0	64.8 ± 8.1	2.271	0.025
BMI (kg/m^2^)	22.77 ± 2.01	23.03 ± 1.95	−0.668	0.505
SOFA score (points)	13.74 ± 1.83	11.52 ± 2.01	5.850	0.000
APACHE II score (points)	23.09 ± 3.46	21.48 ± 3.82	2.237	0.027
ALB (mg/L)	25.74 ± 2.85	27.66 ± 3.07	−3.286	0.001
Mechanical ventilation time (d)	6.1 ± 1.7	5.7 ± 1.9	1.123	0.264
ICU length of stay (d)	10.6 ± 2.1	9.8 ± 1.8	2.092	0.039
Number of MODS (pcs)	3.93 ± 0.87	2.54 ± 0.82	8.379	0.000
MAP (mmHg)	44.62 ± 6.04	52.70 ± 5.51	−7.131	0.000
24 h urine output (mL)	4.81 ± 1.66	6.82 ± 2.20	−5.188	0.000
Gender (%)			0.844	0.356
Male	30 (62.5)	30 (53.57)		
Female	18 (37.5)	26 (46.43)		
Smoking (%)			1.292	0.256
Yes	17 (35.42)	26 (46.43)		
No	31 (64.58)	30 (53.57)		
Drinking (%)			0.504	0.478
Yes	14 (29.17)	20 (35.71)		
No	34 (70.83)	36 (64.29)		
Infection site (%)			9.234	0.026
Intracranial infection	14 (29.17)	6 (10.71)		
Lung infection	17 (35.42)	15 (26.79)		
Blood infection	11 (22.92)	20 (35.71)		
Other	6 (12.5)	15 (26.79)		
Reason for admission to ICU (%)			3.568	0.059
Internal medicine	22 (45.83)	36 (64.29)		
Surgical disease	26 (54.17)	20 (35.71)		

**Table 3:** Logistic regression analysis results.

Index	*β*	SE	Wald's	*P*	OR	95% CI	
Age	0.418	0.206	4.117	0.049	1.519	1.014	2.274
SOFA score	0.592	0.248	5.698	0.017	1.808	1.112	2.939
APACHE II score	0.577	0.265	4.741	0.044	1.781	1.059	2.993
ALB	−0.381	0.264	2.083	0.162	0.683	0.407	1.146
ICU length of stay	0.429	0.257	2.786	0.127	1.536	0.928	2.541
Number of MODS	0.648	0.241	7.230	0.000	1.912	1.192	3.066
MAP	−0.427	0.223	3.666	0.098	0.652	0.421	1.010
24 h urine output	0.331	0.198	2.795	0.126	1.392	0.945	2.053
Intracranial infection	0.727	0.241	9.100	0.000	2.069	1.290	3.318
Day 3 Pcv-aCO2	0.614	0.258	5.664	0.018	1.848	1.114	3.064
Day 3 Pcv-aCO2/Ca-cvO2	0.577	0.259	4.963	0.041	1.781	1.072	2.958
Day 3 blood lactate	0.496	0.237	4.380	0.047	1.642	1.032	2.613
Constant term	1.402	0.618	5.147	0.038	4.063	1.210	13.644

The article "Relationship between Dynamic Changes of Microcirculation Flow, Tissue Perfusion Parameters, and Lactate Level and Mortality of Septic Shock in ICU" was published in 2022. Journal: Contrast Media Mol Imaging.

**Table 4:** ROC curve analysis results.

Index	Sensitivity (%)	Specificity (%)	*P*	AUC	95% CI	
					Lower limit	Upper limit
Day 3 Pcv-aCO_2_	93.72	83.09	0.000	0.943	0.902	0.983
Day 3 Pcv-aCO_2_/Ca-cvO_2_	81.63	77.56	0.000	0.887	0.824	0.949
Day 3 blood lactate	71.66	82.09	0.000	0.825	0.741	0.908

## Data Availability

The raw data supporting the conclusions of this article will be made available by the authors, without undue reservation.
